The article "Circular RNA hsa_circ_0013958 Functions as an Oncogenic Gene Through Modulating miR-532-3p/WEE1 Axis in Hepatocellular Carcinoma" was retracted in 2024. Reasons: original data or images not available; unreliable results or conclusions; concerns about the data.

# Circular RNA hsa_circ_0013958 Functions as an Oncogenic Gene Through Modulating miR-532-3p/WEE1 Axis in Hepatocellular Carcinoma

**DOI:** 10.3389/fonc.2021.585172

**Published:** 2021-04-15

**Authors:** Tao Ma, Yue Ma, Yongjun Du, Zhongheng Wei, Jianchu Wang, Yufu Jun, Fenqiang Xiao

**Affiliations:** ^1^ Department of Clinical Laboratory, Hospital of Chengdu University of Traditional Chinese Medicine, Chengdu, China; ^2^ Department of Gastroenterology, Hospital of Chengdu University of Traditional Chinese Medicine, Chengdu, China; ^3^ Department of Proctology, Hospital of Chengdu University of Traditional Chinese Medicine, Chengdu, China; ^4^ Department of Oncology, Affiliated Hospital of Youjiang Medical University for Nationalities, Baise, China; ^5^ Department of Hepatobiliary Surgery, Affiliated Hospital of Youjiang Medical University for Nationalities, Baise, China; ^6^ Department of Gastroenterology, Shanghai Songjiang District Central Hospital, Shanghai, China; ^7^ Department of Emergency Surgery, Union Hospital, Tongji Medical College, Huazhong University of Science and Technology, Wuhan, China

**Keywords:** hepatocellular carcinoma, circ0013958, miR-532-3p, WEE1, ceRNA

## Abstract

**Background:**

circ0013958 was identified as a biomarker, which can be used for the diagnosis and screening of lung cancer. However, the role of circ0013958 in hepatocellular carcinoma (HCC) remains unclear.

**Methods:**

In our study, quantitative real-time polymerase chain reaction was performed to determine the levels of circ0013958 in HCC tissues and cell lines. EdU, CCK-8, transwell, flow cytometry and tumorigenesis assays were applied to assess the functions of circ0013958 in HCC *in vitro* and *in vivo*. Western blot assay was to detect the expression of WEE1. Luciferase reporter assay, bioinformatics analysis and rescue experiments were used to examine the interaction among circ0013958, miR-532-3p and WEE1.

**Results:**

It revealed that circ0013958 was significantly up-regulated in HCC, which was positively correlated with poor prognosis of HCC patients. Circ0013958 promoted HCC cell proliferation and invasion, inhibited cell apoptosis *in vitro*, and promoted tumorigenesis *in vivo*. Circ0013958 acted as a miR-532-3p sponge to regulate WEE1 expression, thus promoting the progression of HCC.

**Conclusions:**

Circ0013958 promotes HCC progression through miR-532-3p/WEE1 axis. Circ0013958 may serve as a potential diagnostic biomarker and therapeutic target of HCC.

## Introduction

Liver cancer is a major contributor to the worldwide cancer burden, and hepatocellular carcinoma (HCC) accounts for 75–85% of the primary liver cancer. Incidence rates of HCC have increased in many countries in recent decades (1, 2). It ranks as the fourth most common cause of cancer-related death worldwide, with about more than 800,000 new cases and 750,000 deaths (3–5). Contrary to the downward trend in the burden of other cancer diseases, the burden of liver cancer increases over time. Though systemic therapy has markedly developed, the incidence and death rate of HCC still rose over the past decade (6). The complexity of HCC treatments lies in its considerable phenotypic and molecular heterogeneity (7, 8). Therefore, it is urgent that we gain more knowledge about the molecular mechanisms in HCC initiation and development.

A poorly characterized component of the HCC transcriptome is circular RNA (circRNAs), which have been confirmed in recent studies (9–11). Circular RNAs (circRNAs), a novel class of endogenous noncoding RNAs, have a covalently closed circular conformation and are structurally stable (12). Previous studies revealed that circRNAs can compete together with microRNAs (miRNAs) and are involved in biological processes including tumor cell proliferation, apoptosis, invasion, and migration (13–15). For example, circFAT1 promotes HCC progression by sponging miR-30a-5p, Therefore, the advantage of circRNAs as novel biomarkers and therapeutic targets are increasingly becoming clear.

circ0013958 was identified as a potential non-invasive biomarker through RNA sequencing, and thus may contribute to detecting and screening lung cancer (16). However, the role of circ0013958 in HCC remains unclear.

In this present study, we found that 1) circ0013958 was upregulated in HCC tissues and cell lines. 2) circ0013958 promoted cell proliferation, migration and inhibit cell apoptosis in HCC; 3) circ0013958 functioned as a miR-532-3p sponge and regulated WEE1 expression, thus promoting the development of HCC; 4) circ0013958 promoted tumor growth in HCC.

## Materials and Methods

### Tissues and Cell Lines

30 HCC tissues and 25 normal tissues were obtained from the Chengdu University of Traditional Chinese Medicine. All patients assigned their informed consent before this study start. This study was approved by the ethics committee of the Chengdu University of Traditional Chinese Medicine.

293T cells and LO2 cells and HCC cell lines (HepG2, Huh7 and Hep3B) were supplied by the Cell Bank of Type Culture Collection of the Chinese Academy of Sciences (Shanghai, China) and cultured in DMEM media containing 10% fetal bovine serum (Gibco, USA) and 1% penicillin–streptomycin (Gibco, USA) under 5% CO_2_ at 37°C.

### Total RNA Isolation and qRT-PCR

The isolation of total RNA from the cell lines and tissues was performed using TRIzol reagent (Invitrogen, USA) according to the manufacturer’s instructions. Reverse transcription was performed by a high-quality cDNA reverse transcription kit (Thermo Fisher Scientific, USA). The quantitative real-time polymerase chain reaction (qRT-PCR) was performed using SYBR Green Mix (TaKaRa Biotechnology, Japan) and run on an ABI 7900 system (Applied 140 Biosystems, USA). GAPDH and U6 were used as endogenous references. The relative expression of RNA was calculated according to 2^−ΔΔCT^ algorithm. All primers used in this study were listed in **Table S1**.

### Cell Counting Kit-8 Proliferation Assay

Some 100 μl Hep3B and Huh7 cells (3 × 10^3^/ml) were seeded into 96-well plates. After 2 h, added 10 μl CCK-8 reagent (Abcam, USA) to each well and incubated for 2 h. Then the OD value was measured at wavelength of 450 nm using a Multiskan FC with Incubator (Thermo Fisher Scientific, USA).

### 5-Ethynyl-2′-Deoxyuridine (EdU) Assay

Cell proliferation was also evaluated using an EdU assay kit (Ribobio, China). Some 100 μl Hep3B and Huh7 cells (2 × 10^5^) were cultured in 96-well plates and then incubated with 50 μM EdU reagent for 2 h. Then, cells were fixed using 4% paraformaldehyde and staining with DAPI solution. Finally, EdU positive cells were imaged by fluorescence microscopy (Olympus, Japan).

### Transwell Assays

The transwell chambers (Corning, USA) were paved with matrigel mix for invasion assays. HCC cells (2 × 10^5^) were seeded into the upper chambers and cultured in 1 ml medium without fetal bovine serum. Then 2 ml medium containing 10% FBS was added into the to bottom chambers. After 24 h cultivation under 5% CO_2_ at 37°C, the cells in upper chamber were fixed by 4% paraformaldehyde for 15 min and strained by crystal violet for 15 min. The invasive cells were imaged by microscopy.

### Flow Cytometry

Hep3B and Huh7 cells (1 × 10^6^) were suspended and washed three times using cold PBS. Subsequently, cells were stained with 5 µl annexin V (AV) and 5 µl propidium iodide (PI) for 15 min. Flow cytometry (BD Biosciences, USA) was used to analyze the rate of apoptosis.

### Western Blot

We used Image Lab (Bio-Rad Laboratories) for western blotting analysis. The membranes were treated with antibodies including anti-WEE1 (dilution 1:1,000; Cell Signaling Technology, USA), anti-GAPDH (dilution 1:1,000; Cell Signaling Technology, USA) and goat antirabbit secondary antibody (dilution 1:5,000; Cell Signaling Technology). A primary antibody overnight was set at a temperature of 4°C, and a secondary antibody every 1 or 2 h at room temperature.

### Xenografts in Mice

A total of 24 female BALB/c athymic nude mice (4 weeks) were included in animal experiments. The mice were randomly divided into four groups: sh-vector group, sh-circ0013958#1 group, OE-vector group, OE-circ0013958 group. To develop the HCC xenograft model, a total of 1.0 × 10^7^ HCC cells transfected with sh-vector, sh-circ0013958#1, OE-vector, OE-circ0013958 vectors were subcutaneously injected into mice. After 4 weeks, all mice were sacrificed, the weight and volume of tumors were measured. All the animal experiments and any procedure involving animal experiments abide by the Institutional Animal Care and Use Committee of the Affiliated Hospital of Youjiang Medical University for Nationalities.

### Statistical Analysis

The SPSS 23.0 (IBM, USA) and GraphPad Prism 6 (GraphPad, California) were used for data analysis. Student’s t-test or analysis of variance was conducted for comparison of continuous variables. The survival curves were performed using Kaplan–Meier methods and were compared by log-rank tests. P <0.05 was regarded as statistically significant. The Cancer Genome Atlas (TCGA) database was also applied and analyzed.

## Results

### circ0013958 Is Up-Regulated in HCC and Correlated With Poor Survival

To explore the role of circ0013958 in HCC development, we detected circ0013958 expression in HCC tissues and normal tissues by qRT-PCR. It’s found that circ0013958 levels were significantly increased in HCC tissues compared with circ0013958 levels in normal tissues (**Figure 1A**). As shown in **Figure 1B**, circ0013958 levels in HCC cell lines were higher than that in LO2 cells. In addition, it’s found that up-regulated circ0013958 is positively associated with poor prognosis (**Figure 1C**). We also explored TCGA data and found that patients with high expression of ACP6 (the parental gene of circ0013958) have shorter survival time (**Figures 1D, E**). These data suggest that circ0013958 was up-regulated in HCC and positively related with poor survival of HCC patients.

**Figure 1:** The expression of circ0013958 in HCC tissues and cell lines. **(A, B)** The expression of circ0013958 in HCC tissues and cell lines (T means tumor tissue; NT means normal tissue). **(C, D)** The patients with high expression of circ0013958 in HCC had poor prognosis and survival. **(E)** The high ACP6 expression in TCGA has a poor survival. (***p < 0.001).

### circ0013958 Promotes HCC Cell Proliferation, Migration and Inhibits Cell Apoptosis

In **Figure 1B**, we found that Huh7 and Hep3B cell lines presented the highest and lowest levels of circ00139585 in three HCC cell lines. Therefore, Huh7 and Hep3B cells were selected for further functional study. We constructed circ0013958 overexpressing and circ0013958 knockdown HCC cells respectively. It’s showed that HCC cells transfected with OE-circ0013958 vector promoted the expression of circ0013958, but HCC cells transfected with sh-circ0013958 vector inhibited the expression of circ0013958 (**Figures 2A, B**). EdU assay revealed that HCC cells transfected with oe-circ0013958 vectors was promoted the proliferation of cells, while circ0013958 knockdown exerted opposite effect (**Figure 2C**). CCK-8 assay also showed that circ0013958 overexpression significantly increased the proliferation of HCC cells, whereas circ0013958 konckdown decreased the proliferation of HCC cells (**Figure 2D**). Transwell assay showed that circ0013958 overexpression promoted the migration of HCC cells, but circ0013958 knockdown inhibited the migration of HCC cells (**Figure 2E**). And flow cytometry assay revealed that circ0013958 overexpression decreased numbers of apoptotic HCC cells, while circ0013958 inhibition increased promoted the apoptosis of HCC cells (**Figure 2F**). All results demonstrated that circ0013958 significantly promoted the proliferation and migration of cells and suppressed the apoptosis of cells in HCC.

**Figure 2:** Circ0013958 promotes HCC cell proliferation, migration and inhibits HCC cell apoptosis *in vitro*. **(A, B)** Relative expression of circ0013958 in constructed Hep3B and Huh7 cells. **(C, D)** EdU proliferation assay and CCK-8 assay was used to examine the proliferation of Hep3B and Huh7 cells with circ0013958 overexpression or circ0013958 knockdown. **(E)** Transwell assay detected the migration of Hep3B and Huh7 cells with circ0013958 overexpression or circ0013958 knockdown. **(F)** Flow cytometry assay was used to determine the apoptosis of HCC cells with circ0013958 overexpression or circ0013958 knockdown. (**p < 0.01, ***p < 0.001).

### miR-532-3p Interacts With circ0013958 in HCC Cells

Subsequently, we found that downstream miRNAs of circ0013958 in HCC cells by Circular RNA Interactome (https://circinteractome.nia.nih.gov/) and circBase (http://www.circbase.org/). Among these miRNAs, it’s showed that miR-532-3p was significantly enriched in both HCC cells by pull-down assay using circ0013958 probes (**Figure 3B**). The possible binding sites between miR-532-3p and circ0013958 were shown in **Figure 3A**. And the luciferase reporter assay showed that miR-532-3p reduced the luciferase activities of circ0013958 WT group not circ0013958 MUT group, suggesting a direct interaction between circ0013958 and miR-532-3p (**Figure 3C**). Then, we explored the role of miR-532-3p in HCC cells. CCK-8 assay and EdU assay showed that miR-532-3p overexpression inhibited cell proliferation in Huh7 cells, and miR-532-3p inhibition promoted the cell proliferation in Hep3B cells (**Figures 3D, E**). Transwell assay also showed that miR-532-3p overexpression inhibited the migration of cells, but miR-532-3p inhibition promoted the cell migration in HCC cells (**Figure 3F**). Flow cytometry assay showed that miR-532-3p overexpression promoted the apoptosis of cells, but miR-532-3p inhibition inhibited the apoptosis of cells in HCC cells (**Figure 3G**). These findings revealed that circ0013958 could interact with miR-532-3p to promote HCC development.

**Figure 3:** MiR-532-3p targets circ0013958 to inhibit HCC progression. **(A)** Schematic illustration of the sequence of circ0013958 with miR-532-3p. **(B)** qRT-PCR detected the expressions of seven different miRNAs in HCC cells supplied with circ0013958 probes. **(C)** The luciferase reporter assay detected detects the luciferase activity of circ0013958 WT/circ0013958 MUT in HCC cells co-transfected with miR-532-3p mimics. **(D, E)** CCK-8 assay and EdU proliferation assay were used to examine the proliferation of HCC cells. **(F)** Transwell assay detected the migration of HCC cells. **(G)** Flow cytometry assay was used to determine the apoptosis of HCC cells. (**p < 0.01, ***p < 0.001).

### MiR-532-3p Interacts With WEE1

We screened targets that may be potentially regulated by miR-532-3p using public available databases including ENCORI (The Encyclopedia of RNA Interactomes, http://starbase.sysu.edu.cn/index.php) and TargetScan (http://www.targetscan.org/vert_72/). It’s found that WEE1 was potential target of miR-532-3p, the possible binding sites between miR-532-3p and WEE1 were shown in **Figure 4A**. TCGA database showed that high WEE1 expression was associated with poor survival (**Figure 4B**). qRT-PCR showed that WEE1 was up-regulated in HCC tissues (**Figure 4C**). Luciferase reporter assay showed that miR-532-3p significantly reduced the luciferase activities in WEE1 WT group not in WEE1 MUT group, suggesting that miR-532-3p could interact with WEE1 in HCC cells (**Figure 4D**). Western blot also showed that miR-532-3p overexpression inhibited the expression of WEE1 in HCC cells, but circ0013958 overexpression could reverse the inhibitory effect of miR-532-3p overexpression on the WEE1 expression (**Figure 6E**). These findings suggest that circ0013958 could interact with miR-532-3p to regulate WEE1 in HCC cells.

**Figure 4:** MiR-532-3p targets WEE1 in HCC. **(A)** Schematic illustration of the sequence of WEE1 with miR-532-3p. **(B)** High WEE1 expression had poor survival in TCGA database. **(C)** The WEE1 expressions in HCC samples by qRT-PCR. **(D)** The luciferase reporter assay detected detects the luciferase activity of WEE1 WT/WEE1 MUT in HCC cells co-transfected with miR-532-3p mimics. **(E)** Western blot detected WEE1 expressions in HCC cells stimulated with NC mimics, miR-532-3p mimics and oe-circ0013958+ miR-532-3p mimics. (***p < 0.001).

### Circ0013958 Promotes HCC Cell Proliferation, Migration and Inhibits Cell Apoptosis by miR-532-3p/WEE1 Axis

Further studies showed that circ0013958 promoted the expression of WEE1 in HCC cells by western blotting (**Figure 5A**). CCK-8 assay and EdU assay (**Figures 5B, C**) showed that circ0013958 knockdown inhibited the proliferation of Huh7 cells, while WEE1 overexpression reversed this effect of inhibitory role of circ0013958 knockdown in Huh7 cells. And circ0013958 overexpression promoted the proliferation of Hep3B cells, while WEE1 knockout reversed this effect of inhibitory role of circ0013958 overexpression in Hep3B cells. In addition, the results of transwell assay and flow cytometry assay also indicated that circ0013958 promoted cell migration and inhibited cell apoptosis in HCC cells (**Figures 5D, E**). These results demonstrated that circ0013958 promoted HCC development by regulating WEE1.

**Figure 5:** Circ0013958 promotes HCC development by miR-532-3p/WEE1 axis. **(A)** Western blot detected WEE1 expressions in HCC cells stimulated with sh- circ0013958, sh-circ0013958 + OE-WEE1, OE-circ0013958, OE-circ0013958 + si-WEE1. **(B, C)** CCK-8 assay and EdU proliferation assay were used to examine the proliferation of HCC cells treated with sh-circ0013958, sh-circ0013958 + OE-WEE1, OE-circ0013958, OE-circ0013958 + si-WEE1. **(D)** Transwell assay detected the migration of HCC cells transfected with sh-circ0013958, sh-circ0013958 + OE-WEE1, OE-circ0013958, OE-circ0013958 + si-WEE1. **(E)** Flow cytometry assay was used to determine the apoptosis of HCC cells transfected with sh-circ0013958, sh-circ0013958 + OE-WEE1, OE-circ0013958, OE-circ0013958 + si-WEE1. (*p < 0.05, **p < 0.01, ***p < 0.001).

### circ0013958 Promotes Tumorigenesis of HCC *In Vivo*

To further investigated the function of circ0013958 *in vivo*, Hep3B cells transfected with oe-circ0013958 and Huh7 cells transfected with sh-circ0013958 were injected into mice, respectively. As shown in **Figures 6A, B**, circ0013958 knockdown inhibited the tumor growth in HCC, while circ0013958 overexpression promoted the tumor growth of HCC. We also found that circ0013958 knockdown promoted the expression of miR-532-3p and inhibited the expression of WEE1, but circ0013958 overexpression inhibited the expression of miR-532-3p and promoted the expression of WEE1 in tumor tissues (**Figures 6C–E**). These results suggest that circ0013958 promoted the tumor growth of HCC *in vivo*.

**Figure 6:** Circ0013958 promotes tumorigenesis of HCC *in vivo*. **(A, B)** Tumor specimens and volume in nude mice that injected with sh-circ0013958 cells and oe-circ0013958 cells. ^©^ The relative expression of circ0013958 in tumors from mice injected with sh-circ0013958 cells and oe-circ0013958 cells. **(D)** The relative expression of miR-532-3p in tumors from mice injected with sh-circ0013958 cells and oe-circ0013958 cells. **(E)** The expression of WEE1 in tumors from mice that injected with sh-circ0013958 cells and oe-circ0013958 cells. (**p < 0.01, ***p < 0.001).

## Discussion

Recently, many studies have revealed the role of circRNAs in cancer progression (17). circRNAs can function as a miRNA “sponge” and therefore provide novel therapeutic treatment for human cancers (18–20). Therefore, circRNAs can downregulate miRNAs and play an important role in cancer development.

Here, we demonstrated that circ0013958 was elevated in HCC. Previous studies found that circ0013958 was up-regulated in adenocarcinoma through tumor-specific circRNA microarrays, as well as associated with TNM stage and lymphatic metastasis (16). However, the role of circ0013958 in HCCs still remains unknown. We found that circ0013958 promoted cell proliferation and inhibited cell apoptosis in HCCs, which was partially in accordance with the function of circ0013958 in lung adenocarcinoma.

circRNAs have been found to act as miRNA sponges in many diseases. We also found that circ0013958 could bind to miR-532-3p, which has been identified to affect cancer tumors development (21–23). Gu et al. reported that miR-532-3p acted as a tumor suppressor in colorectal cancer progression *via* modulating the Wnt/β-catenin axis (24). Feng et al. illustrated that miR-532-3p inhibited tongue squamous cell carcinoma from malignant behaviors by disrupting CCR7 signaling. These studies demonstrated the role of miR-532-3p as a tumor suppressor, which was consistent with our results that miR-532-3p knockdown promote cell proliferation and migration of HCC tumors. Deep studies showed that miR-532-3p can target WEE1 in HCC cells. Tyrosine kinase WEE1 inhibits CDK1/2 to regulate DNA synthesis during S phase, and as a response to DNA damage, can prevent entry into mitosis (25). Overexpressed WEE1 was related to poor survival of breast cancer, colorectal cancer and gastric cancer (26–29).

This study found that that circ0013958 might bind miR-532-3p to modulate the expression of WEE1 in HCC to promote tumor progression, demonstrating the role of circ0013958 as a novel therapeutic target in HCC patients.

There are several limitations in this study, for example 1) because of the shortage of clinicopathological data, we could not explore the association between circ0013958 and TNM stage, as well as tumor grade in HCC though *in vitro* and *in vivo* assays demonstrated that elevated circ0013958 was correlated with poor prognosis; 2) WEE1 inhibitor was not applied in current study, while our western blot results showed the function of miR-532-3p in inhibiting WEE1 expression, which could be rescued by circ0013958.

In brief, this study revealed that circ0013958 was upregulated in HCC patients and was correlated with poor prognosis. Moreover, our study identified the role of circ0013958 as a sponge to miR-532-3p, thus enhancing the expression of oncogenic WEE1 that plays an important role in HCC development. Consequently, we identified circ0013958 might have a potential as a prognostic biomarker and therapeutic target for HCC.

## Data Availability Statement

The original contributions presented in the study are included in the article/**Supplementary Material**. Further inquiries can be directed to the corresponding authors.

## Ethics Statement

The studies involving human participants were reviewed and approved by Chengdu University of Traditional Chinese Medicine. The patients/participants provided their written informed consent to participate in this study. The animal study was reviewed and approved by The Ethics Committee of the Affiliated Hospital of Youjiang Medical University for Nationalities.

## Author Contributions

YJ and FX designed the project. TM, YM, and YD performed the experiments and wrote the manuscript. ZW and JW processed the data. All authors contributed to the article and approved the submitted version.

## Conflict of Interest

The authors declare that the research was conducted in the absence of any commercial or financial relationships that could be construed as a potential conflict of interest.
